The article "The Cellular Distribution of Serotonin Transporter Is Impeded on Serotonin-Altered Vimentin Network" was retracted in 2019. Reasons: manipulated images; duplicated images; original data or images not available.

# The Cellular Distribution of Serotonin Transporter Is Impeded on Serotonin-Altered Vimentin Network

**DOI:** 10.1371/journal.pone.0004730

**Published:** 2009-03-09

**Authors:** Billow A. Ahmed, Irfan A. Bukhari, Brandon C. Jeffus, Justin T. Harney, Sheeno Thyparambil, Endrit Ziu, Mony Fraer, Nancy J. Rusch, Piotr Zimniak, Vladimir Lupashin, Dale Tang, Fusun Kilic

**Affiliations:** 1 Department of Biochemistry and Molecular Biology, College of Medicine, The University of Arkansas for Medical Sciences, Little Rock, Arkansas, United States of America; 2 Department of Internal Medicine, College of Medicine, The University of Arkansas for Medical Sciences, Little Rock, Arkansas, United States of America; 3 Department of Pharmacology, College of Medicine, The University of Arkansas for Medical Sciences, Little Rock, Arkansas, United States of America; 4 Department of Physiology, College of Medicine, The University of Arkansas for Medical Sciences, Little Rock, Arkansas, United States of America; 5 Center for Cardiovascular Sciences, Albany Medical College, Albany, New York, United States of America; Dalhousie University, Canada

## Abstract

**Background:**

The C-terminus of the serotonin transporter (SERT) contains binding domains for different proteins and is critical for its functional expression. In endogenous and heterologous expression systems, our proteomic and biochemical analysis demonstrated that an intermediate filament, vimentin, binds to the C-terminus of SERT. It has been reported that 5HT-stimulation of cells leads to disassembly and spatial reorientation of vimentin filaments.

**Methodology/Principal Findings:**

We tested the impact of 5HT-stimulation on vimentin-SERT association and found that 5HT-stimulation accelerates the translocation of SERT from the plasma membrane via enhancing the level of association between phosphovimentin and SERT. Furthermore a progressive truncation of the C-terminus of SERT was performed to map the vimentin-SERT association domain. Deletion of up to 20, but not 14 amino acids arrested the transporters at intracellular locations. Although, truncation of the last 14 amino acids, did not alter 5HT uptake rates of transporter but abolished its association with vimentin.

To understand the involvement of 5HT in phosphovimentin-SERT association from the plasma membrane, we further investigated the six amino acids between Δ14 and Δ20, i.e., the SITPET sequence of SERT. While the triple mutation on the possible kinase action sites, S_611_, T_613_, and T_616_ arrested the transporter at intracellular locations, replacing the residues with aspartic acid one at a time altered neither the 5HT uptake rates nor the vimentin association of these mutants. However, replacing the three target sites with alanine, either simultaneously or one at a time, had no significant effect on 5HT uptake rates or the vimentin association with transporter.

**Conclusions/Significance:**

Based on our findings, we propose that phosphate modification of the SITPET sequence differentially, one at a time exposes the vimentin binding domain on the C-terminus of SERT. Conversely, following 5HT stimulation, the association between vimentin-SERT is enhanced which changes the cellular distribution of SERT on an altered vimentin network.

## Introduction

The serotonin transporter (SERT) is a member of a larger family of Na^+^- dependent transporters in prokaryotes and animals, which is designated the SLC6 or NSS family. The biogenic amine transporter family shares about 60% amino acid identity overall [1]–[4]. SERT exists as a 630 amino acid plasma membrane bound glycoprotein in which both the amino (N) and carboxyl (C) termini are cytosolic.

The termini domains of monoamine transporter proteins have garnered significant attention for their importance in transport function and localization. Several proteins have been identified in association with the C-terminus of SERT such as PICK1 [5]–[7], the actin cytoskeleton [8], neuronal nitric oxide synthase, Sec23A, Sec24C (5), fibrinogen, an activator of integrin αIIbβ3 [9]. Additionally, the interaction with MacMARCKS has been shown to modulate 5HT uptake, endocytosis, and phosphorylation of SERT via activating protein kinase C (PKC) [10] in a biphasic manner [11]. Studies have also shown that PKC-dependent modulation of SERT is correlated with extracellular 5HT levels [12], [13]. More specifically, it has been suggested that the final 20 amino acids of the C-terminal of SERT are critical for the functional expression of the transporter [14], [15].

Our recent findings explained the role of the C-terminus in the localization and trafficking of SERT via Rab4 a small GTPase, in a plasma 5HT-dependent manner. These studies demonstrated that elevated plasma 5HT “paralyzes” the translocation of SERT from intracellular locations to the plasma membrane by controlling transamidation and Rab4-GTP formation [15].

In endogenous, platelet system, we have also observed the biphasic effect of plasma 5HT on platelet SERT [16]. More specifically, in the serum of prehypertensive subjects in which the plasma 5HT level was slightly higher than physiological levels, 5HT uptake rates and the density of SERT on the platelet plasma membrane were found significantly higher than those on platelets from normotensive states [16]. However, in plasma of hypertensive subjects in which 5HT concentration was further elevated, the 5HT uptake rates of SERT was low due to a decrease in the number of the transporters on the platelet plasma membrane [16]. Importantly, neither the mediators playing a role in 5HT-dependent regulation of SERT density on the plasma membrane nor the mechanism by which they are effective on SERT density as a factor of plasma 5HT-levels have fully been identified yet.

In a series of previously reported experiments, it was found that 5HT-stimulation of cells activates p21 activating kinase (PAK), which in turn phophorylates vimentin on the serine residue at position 56 [17]. Following phosphorylation, the curved filamentous structure of vimentin undergoes reorganization and straightens [18]. Therefore, as reported here, we analyzed the vimentin-SERT association in platelets and then explored the role of plasma 5HT on this association, i.e., whether the disassembly and spatial reorganization of the vimentin network affects the translocation and, in turn, the cellular distribution of SERT molecules. Our biochemical and proteomic analysis of the proteins associated with the C-terminus of SERT identified vimentin, an intermediate filament in between many other platelet proteins.

Based on our studies detailed here, we propose that phosphate modification of the SITPET sequence of SERT one at a time exposes the C-terminus domain of SERT for vimentin association. Conversely, following 5HT stimulation, the association between vimentin-SERT is enhanced specifically on the plasma membrane which controls the cellular distribution of SERT on an altered vimentin network.

## Materials and Methods

### Plasmids, constructs, and cell line expression systems

Human SERT (hSERT) tagged on its amino terminus with yellow fluorescent proteins (YFP) was studied for the specificities previously and no significant differences between the 5HT uptake efficiencies of tagged or wild-type hSERT were observed [15].

The mutant transporters were constructed utilizing a Stratagene Quickchange XL site-directed mutagenesis kit. The primer sequences are listed in Table S1. All synthetic constructs were verified via DNA sequencing.

Cells were grown, and transfection was achieved, as described previously [19]. To test the impact of 5HT on cellular SERT system, transfected cells were pretreated with 5HT for 30-min at room temperature (RT) and then the assays were performed.

### Immunofluorescent (IF) analysis

IF imaging cells grown on glass coverslips to 50–60% confluence in 35-mm dishes were transfected with the respective plasmids, fixed, stained and imaged after 24 h. We used the 63× oil 1.4 numerical aperture (NA) objective of a LSM510 Zeiss Laser inverted microscope outfitted with confocal optics for image acquisition. Subsequent scanning for each individual channel was performed. YFP was exited at 488 nm with Argon2 laser and emission was recorded through a 500–530-nm infrared band-pass filter. Texas Red fluorescence was excited at 543 nm with a helium-neon laser, and the emitted light was recorded through a 560-nm long-pass filter. Single *z*-sections were collected (0.8 μm thick) using Zeiss LSM 510 software (Release Version 4.0 SP1). Images were cropped with Adobe Photoshop 6.0 software.

### 5HT Uptake Assay

Transport assays were performed in 24 well plates at RT. Twenty-four hours after transfection, cells were washed with phosphate-buffered saline (137 mM NaCl, 2.7 mM KCl, 4.3 mM Na_2_HPO_4_, and 1.4 mM KH_2_PO_4_, pH 7.3) (PBS) containing 0.1 mM CaCl_2_ and 1 mM MgCl_2_ (PBS/CM). Transport was measured by incubating the cells in 250 μl of PBS/CM containing the radio-labeled substrate (1,2-^3^H(N))5HT (14.6 nM final concentration; specific activity) 20.5 Ci/mmol (New England Nuclear, Inc., Boston, MA; #NET-498) for 10 min at RT, an interval previously determined to include only the initial, linear phase of the transport. Each well was washed very quickly three times with ice-cold PBS. The cells were lysed in 100 ml of 1% SDS and each well's contents were transferred to a scintillation vial and counted in 3 ml of Scintisafe Econo1 (Fisher Scientific, Pittsburgh, PA) [19].

Background accumulation of (^3^H)-serotonin was measured in the same experiment using mock-transfected cells and subtracted from each experimental value. Maximum background accumulation was 0.01 pmol/mg protein/min. All determinations were performed at least in triplicate. Data were then plotted using OriginLab 7.5 (Northampton, MA), and statistical analyses were conducted using the NCSS software package (Number Cruncher Statistical Systems, Kaysville, UT). Analysis of variance (ANOVA) was used to determine whether mutations or deletions changed transport activity significantly relative to control or according to cell line. P-values were adjusted for multiple comparisons using either Dunnett's or Bonferroni correction procedures.

### Peptide-Affinity Chromatography and Mass Spec Analysis

To identify platelet proteins that interact with the C terminus of SERT, we used a proteomic approach based on peptide affinity chromatography by using a synthetic peptide corresponding to the last 26 amino acids from the C-terminus (586–630) of SERT. Proteintech Group, Inc. (Chicago, IL) synthesized the peptide and conjugated to GST Sepharose beads. GST was used as an arm between peptide and Sepharose to increase the distance between peptide and matrix to facilitate the interaction between peptide and the cytosolic protein in the cell lysate. Our control column was 3 ml of GST-Sepharose without peptide. Once we set the peptide-affinity column, the platelets were isolated and the soluble proteins were prepared to run on column.

Platelets were isolated from 20 ml blood samples and lysed. 1.0% TX-100 soluble lysates were loaded on control GST columns and GST-peptide columns. The proteins bound to the columns were eluted using 500 mM NaCl and fractions were collected. The peak fractions were pooled and concentrated on microfilterfuge tubes with a 10 kD cut off (Rainin Instrument Co., Oakland, CA). The concentrated samples were resolved by SDS-PAGE. Two major bands appeared in the peptide-GST Sepharose column but did not appear in our control, the GST-Sepharose column.

The 115 and 60 kD bands were eluted and processed robotically using a ProGest instrument (Genomic Solutions), as previously described [20]. The resultant 50 ml peptide pools were analyzed using nano LC/MSMS on a LCQ Deca XP Plus ion trap mass spectrometer.

### Western Blot (W/B) Analysis

Cells were solubilized in PBS containing 0.44% SDS, 1 mM phenylmethylsulfonyl fluoride (PMSF), and protease inhibitor mixture (PIM). The PIM, which contained 5 μg/ml pepstatin, 50 μg/ml leupeptin, and 5 μg/ml aprotinin, was included with each lysis buffer [19]. Samples were analyzed by SDS-PAGE and transferred to a nitrocellulose membrane. SERT was detected by using SERT monoclonal antibody (MAb Technology, Stone Mountain, GA) (diluted 1:400) and HRP-conjugated anti-mouse IgG (diluted 1:5,000). The signal was visualized by using an enhanced chemiluminescence W/B detection system (Pierce, Rockford, IL). The polyclonal SERT antibody was purchased from Chemicon International (Temecula, CA; catalog number: AB1594P).

In W/B analysis, PAK-phosphorylation of vimentin was detected with a specific vimentin Ser-56 (pS56) antibody (Ab) [17], [18]. pS56-Ab was prepared against a synthetic phosphopeptide (Ser-Leu-Tyr-Ala-Ser-phosphoSer56-Pro-Gly-Gly-Ala-Tyr-Cys) by SynPep Inc. (Dublin, CA). Using standard affinity purification procedures, pS56A Ab was purified on Protein A Sepharose column [21]. Vimentin-Ab (Research Diagnostics, Inc. Concord MA) reacts with vimentin and phosphovimentin dually; in contrast, phosphovimentin-(pS56)-Ab reacts only with phosphovimentin [17].

### Cell surface biotinylation

Cell surface expression of the transporters was detected after biotinylation with the membrane-impermeant biotinylation reagent sulfo-NHS-SS-biotin, as described previously [15], [19]. Briefly, cells were treated with 100 mM glycine to complete quenching of the unreacted NHS-SS-biotin and lysed in TBS containing 1% SDS, 1% TX100, and PIM/PMSF. The biotinylated proteins (500 μl) were recovered with an excess amount of streptavidin-agarose beads (400 μl) after overnight incubation. After biotinylated proteins were eluted in 100 μl sample buffer and separated on SDS-PAGE, they were transferred to nitrocellulose and were detected with anti-SERT antibody, as described [19].

Densitometric scanning of W/B was done on VersaDoc digital imaging system (BioRad). On each gel, samples were compared with the biotinylation procedure applied to the same amount of cells as determined by the BCA protein assay (Pierce, Rockford, IL). The experiments were performed within the linear range of densitometry reading of the SERT band as a function of the amount of protein applied according to control experiments with varying amounts of protein load per lane. Densitometry data were captured as total signal in the rectangular area encompassing the band of study corrected for background; the same rectangular area was used for estimates of the same band in other lanes of gel. Results from different scans were uniform.

## Results

### Vimentin and phosphovimentin associate with SERT in platelets

A synthetic peptide corresponding to the last 26 amino acids from the C-terminus (586–630) of SERT was conjugated to GST Sepharose beads. As described in the Methods section, the GST was used as an arm between the peptide and Sepharose to increase the distance between the peptide and matrix to facilitate the interaction between the peptide and the cytosolic protein in the cell lysate. Detergent solubilized platelet lysate was run on the peptide-affinity column. The proteins bound to the columns were eluted and concentrated on microfilterfuge tubes with a 10 kD cut off. The concentrated samples were resolved by SDS-PAGE (data not presented). Two major 115 and 60 kD bands appearing in the peptide-GST but not control GST-column were eluted, processed, and analyzed using nano LC/MSMS on a LCQ Deca XP Plus ion trap mass spectrometer as previously described [20]. Our proteomic approach identified vimentin as one of many platelet proteins bound to the C-terminus of SERT. Furthermore, we analyzed these findings with biochemical techniques following the endogenous expression of vimentin and SERT in platelets with W/B assays (Fig. 1A). The co-IP assays agreed with our ESI-MS/MS mass spectrometry result showing the association between vimentin and SERT in platelet (Fig. 1B and C).

**Figure 1:** SERT and vimentin interaction in human platelets. *(A)* Endogenous vimentin and SERT expression in platelets were analyzed with W/B analysis. The association between vimentin and SERT was determined by a co-IP in platelets stimulated with 0, 1, and 2 nM 5HT. Following 5HT-stimulation, platelet lysate was divided into two portions; the half portion of lysate was incubated in anti-vimentin monoclonal Ab *(B)*, the other half portion in anti-SERT Ab coated protein A Sepharose beads *(C)*. Next day, vimentin- or SERT-Ab pulled down proteins were eluted from sepharose beads; both IP eluents were analyzed either with a polyclonal SERT Ab, or with pS56-Ab, respectively. Nonspecific adsorption of Sepharose beads was not determined in the absence of antibodies. The association between endogenous vimentin and SERT was altered in a 5HT concentration-dependent manner. The highest amount of SERT was pulled down by vimentin-Ab in 2 nM 5HT-stimulated platelets. Additionally, vimentin associated with SERT after 2 nM-5HT stimulation was in phosphorylated form. *(D)* Expression of SERT and vimentin in total cell lysates was determined by W/B analysis as a loading control. All lanes contain protein recovered from the same number of platelets (1.5×10^8^). Figures show representative images from 2 to 4 separate experiments.

It is reported that stimulation of cells with 5HT induced phosphorylation of vimentin on serine at position 56, resulting in the reorganization of the vimentin network [17], [18]. Consequently, we investigated the impact of 5HT stimulation on vimentin-SERT association. Platelets in platelet poor plasma (PRP) were first stimulated with 1 or 2 nM 5HT, which represents the plasma levels of 5HT in normotensive and hypertensive patients, respectively, and thus a physiologically relevant stimulus [16]. Following a 30-min pretreatment with 5HT at RT, platelets were pelleted, lysed in IP-lysing buffer, and precleared [19]. The platelet lysate was divided into two half portions. The IP assay was performed on both portions using either a monoclonal vimentin-Ab or monoclonal SERT-Ab.

The proteins precipitated on vimentin-Ab were subjected to immunoblot analysis using anti-SERT Ab (Fig. 1B). The level of SERT on vimentin-Ab was increased in a 5HT concentration-dependent manner. Stimulation of platelets with 2 nM 5HT enhanced SERT-vimentin association in whole platelet significantly (Fig. 1B).

Since 5HT-stimulation of cells leads to the phosphorylation of vimentin on the Serine56 residue which alters the filamentous structure of this cytoskeletal protein [17], [18], the reorganization of the vimentin network should regulate the translocation of proteins that utilize the vimentin network [18]. Therefore, we next evaluated the impact of 5HT stimulation on SERT-phosphovimentin association in order to understand the involvement of phosphovimentin in the translocation process of SERT.

We then analyzed the proteins precipitated on SERT-Ab by W/B using a polyclonal phosphovimentin-(pS56)-Ab, which reacts only with the phosphovimentin (Fig. 1C). In contrast, vimentin-Ab dually reacts with vimentin and phosphovimentin [17].

pS56-Ab identified a major band around 55 kD only in 2 nM 5HT pretreated platelet lysate. Thus, these data demonstrate the presence of an association between SERT and phosphovimentin (Fig. 1C).

Therefore, the level of association between vimentin and SERT in Fig. 1B and C represents the total intracellular and plasma membrane. Overall, these findings show that vimentin associates with SERT in an endogenous system, the platelet. Their association was not due to 5HT-dependent stimulation of the platelet; even in the unstimulated form, vimentin-SERT association can be detected (Fig. 1B). However, when the level of 5HT was increased to 1 nM, the precipitated amount of vimentin on SERT was also elevated; therefore, 5HT enhances vimentin-SERT association (Fig. 1B). In the presence of 2 nM 5HT when vimentin is phosphorylated, a high affinity association between SERT and phosphovimentin was observed (Fig. 1C). Additionally, the levels of vimentin and SERT in the whole platelet lysate were not altered at different 5HT concentrations (Fig. 1D).

Since the co-IP assays demonstrated that 5HT-stimulation enhanced the association between vimentin and SERT in platelets, we next addressed (i) whether their association was limited to intracellular locations or also occurred on the plasma membrane; (ii) whether 5HT-dependent elevation of phosphovimentin-SERT association also occurred on the plasma membrane. We performed surface biotinylation followed by W/B assays on platelets stimulated with different concentrations of 5HT.

### Vimentin and phosphovimentin associate with SERT on platelets plasma membrane

To determine the involvement of phosphovimentin in the density of SERT on platelet plasma membrane, platelets in PRP were first pretreated with 5HT (0–2 nM) for 30 min at RT, then the pelleted platelets was biotinylated with membrane impermeable NHS-SS-biotin [16]. Biotinylated platelet plasma membrane proteins were retrieved on streptavidin beads and eluted from the beads.

Half of each biotinylated sample was subjected to immunoblot analysis using anti-SERT Ab (Fig. 2A). The biphasic effect of plasma 5HT on the density of SERT on platelet plasma membrane was observed, as seen previously in hypertension model systems [16]. An intermediate level (1 nM) 5HT-stimulation increased the density of SERT on the platelet; however, at high level (2 nM), 5HT-stimulation lowered the surface density of SERT compared to untreated platelets [15], [16].

**Figure 2:** Effect of 5HT stimulation on SERT-vimentin association on platelet plasma membrane. 0–2 nM 5HT-stimulated platelets were biotinylated with NHS-SS-biotin [15], [16], [19], and biotinylated plasma membrane proteins were retrieved on streptavidin beads. Half of biotinylated platelet membrane proteins were analyzed for SERT *(A)*, and the other half was analyzed for anti-phosphovimentin-Ab (pS56-Ab) *(B)* with W/B. Neither SERT not pS56-Ab detected recognizable proteins in mock biotinylated controls (carried through the biotinylation procedure without the addition of the biotinylation reagent); therefore, they are not presented in the blots. Plasma 5HT levels had a biphasic effect on the plasma membrane expression of platelet SERT [16]. To correlate SERT-phosphovimentin association on the surface density of platelet SERT, the biotinylated platelet membrane proteins were analyzed with pS56-Ab. Plasma 5HT, only at high level, showed an association between phosphovimentin-SERT. Intracellular SERT *(C)* and vimentin *(D)* were determined by W/B analysis of non-bound material and also served as a loading control. All lanes contain protein recovered from the same number of platelets (1.5×10^8^). Figures show representative images from 3 separate experiments.

Here, our data demonstrate that the association between SERT and vimentin is altered in a 5HT-dependent manner. Therefore, here we tested whether the cellular distribution of SERT is altered by 5HT-dependent phosphorylation of vimentin. The level of phosphovimentin on the plasma membrane 5HT-stimulated platelet was evaluated.

The other half of the biotinylated platelet plasma membrane proteins was subjected to immunoblot analysis with pS56-Ab (Fig. 2B). Phosphovimentin appeared as one of the proteins associated with biotinylated plasma membrane-bound proteins in 5HT-stimulated platelets.

SERT could be one of the other phosphovimentin-associated membrane proteins, but our co-IP data in 5HT-stimulated platelets also demonstrated an elevation in the association of SERT-phosphovimentin in whole platelet (Fig. 1C). Therefore, we tested SERT-phosphovimentin association in 5HT-stimulated platelets.

The effects of 5HT-stimulation on the amount of intracellular SERT (flow through of the streptavidin beads) mirrored those of the cell surface SERT (Fig. 2C and D).

Previously, it has been shown that 5HT-stimulation phosphorylates vimentin on the Serine56 residue, but the vimentin S56A mutant is not phosphorylated by 5HT-stimulation [18]. Therefore, to mechanistically determine how the vimentin-SERT association responds to 5HT for regulating the distribution of transporter molecules between plasma membrane and intracellular locations, the S56A mutant and the C-terminus truncated forms of SERT were studied in a CHO heterologous expression system. Obviously, not all aspects of 5HT biology in platelets can be recapitulated in CHO cells, but the CHO model system allows for the analysis of the association between vimentin and the C-terminus truncated forms of SERT and the nonphosphorylated mutant form of vimentin S56A.

To ascertain the optimal 5HT concentration required to stimulate CHO cells expressing hSERT (CHO-hSERT), we measured the density of SERT proteins on the plasma membrane of CHO-hSERT cells and compared this finding to human platelet membranes using biotinylation [15]. In this previous study, we tried to model the effect of plasma 5HT on platelet SERT in a heterologous expression system. Simply stated, an equal amount of biotinylated membrane proteins from CHO-SERT cells and platelets were resolved and analyzed by W/B using SERT-Ab. These calculations together with the dose response analysis of CHO cells to 5HT-stimulation which was already conducted in our previous studies showed that the expression of SERT on the plasma membrane of CHO-SERT cells was 59-fold higher than on the platelet membrane [15]. This estimation indicated that the effect of plasma 5HT at a concentration of 1 nM on platelet SERT may correspond to exogenous 5HT at a concentration of ∼45 μM on CHO-SERT cells [15].

### Co-localization of Vimentin and SERT with or without 5HT stimulation

For the current study, we took a second approach for testing the association between phosphovimentin and SERT on the plasma membrane of 5HT-stimulated cells.

The co-localization of the red vimentin and green YFP-SERT signals were captured in the overlaid images with YFP and Texas Red filter sets. If vimentin and SERT co-localized then the structures would appear light orange; otherwise, the distinct green and red signals would represent structures containing either one of the two proteins. Fifty cells were examined for colocalization of vimentin and SERT following 5HT stimulation. In all YFP-SERT transfected cells, a limited but consistent co-localization between vimentin and SERT on the plasma membrane was seen (Fig. 3).

**Figure 3:** Vimentin-SERT co-localization and impact of 5HT-stimulation on their cellular distribution. CHO-YFP-SERT cells were pretreated with 5HT as indicated, labeled with vimentin monoclonal Ab, and stained with Texas Red conjugated rabbit IgG. In unstimulated cells, vimentin revealed curved filamentous structures; in 5HT-stimulated ones the vimentin filaments became straight as indicated with arrows. Cells were analyzed with a Zeiss LSM510 laser confocal microscope. To contrast the localization of SERT and vimentin, the overlaid images are presented with SERT signal pseudocolored in green. The bar (10 μm) indicates the magnification of the main figures; the insets are 2× the magnification of the main figures. Figures show representative images from at least 2 separate experiments.

The colocalization of endogenously expressed vimentin and transiently expressed SERT was monitored in 5HT-stimulated CHO-(YFP-SERT) cells using IF microscopy. The cellular distribution of vimentin was significantly different in 5HT-stimulated cells than in control cells. To facilitate a comparison between the localization of SERT and vimentin, the SERT signal was pseudocolored in green in merged images. 5HT stimulation mostly located vimentin around the plasma membrane. Exposure of CHO-YFP-hSERT to 5-HT induced the spatial reorientation of vimentin filaments (Fig. 3). In control cells, vimentin exhibited a curved filamentous appearance (Fig. 3, control panel, insert). Vimentin filaments became more straight and bundled 30 min after stimulation with 100 μM 5HT (Fig. 3, 5HT-treated cells panel, insert).

### Vimentin binding domain on the C-terminus of SERT

The C-terminus of the biogenic amine transporter plays a critical role in the regulation of transporter function and intracellular trafficking [5]–[15]. Our proteomic studies identified the C-terminus of SERT as a vimentin binding domain on SERT. To map the vimentin binding sequence on the C-terminus of SERT, we utilized the truncated form of transporters, Δ26, Δ20, Δ14, and Δ6 [15]. As we reported in a previous study, the 5HT uptake rates and the levels of surface expression of Δ6 and Δ14 of SERT were similar to the wild-type transporter [15]. These results were not due to altered protein translation as evident by W/B and densitometry analysis showing that the band densities of all constructs were similar [15].

Next, the association between endogenously expressed vimentin and transiently expressed truncated forms of transporters were tested in 5HT-stimulated CHO cells with IP analysis (Fig. 4). The cellular proteins on the vimentin-Ab coated protein A beads were eluted and separated on SDS-PAGE followed by immunoblotting with SERT-Ab (Fig. 4). The major band at 90 kD was detected in the CHO-SERT and -Δ6 cells (Fig. 4).

**Figure 4:** Vimentin binding domain on the C-terminus of SERT. CHO cells expressing the indicated SERT constructs were lysed and prepared for IP. The cell lysate was incubated with monoclonal anti vimentin-Ab coated protein A sepharose beads. The presence of SERT truncations was detected with a polyclonal SERT Ab (Chemicon International). Since SERT-Δ6 bound to vimentin and the other truncations, we proposed that the amino acids 616–624 are at least one of the vimentin binding domains on the C-terminus of SERT. Nonspecific adsorption of Sepharose beads was not determined in the absence of vimentin-Ab and the data obtained from this set of experiment is not presented here since it can be found in Figure 1B. All lanes contain protein recovered from the same number of cells equivalent to 30% of one well from a confluent 24-well culture plate. Figure shows representative images from 3 separate experiments.

Our recent study compared the distribution of these truncated YFP-SERT variants with that of Texas Red conjugated wheat germ agglutinin (WGA), a lectin marker for the plasma membrane [15]. The IF analysis and 5HT uptake rates showed a lack of colocalization between Δ26 and Δ20 and plasma membrane [15]. Although deletion of up to 20, but not 14 amino acids arrested the transporters at intracellular locations [15], Δ14 like the other two mutants, Δ20 and Δ26, did not co-IP with vimentin (Fig. 4). These data identify the residues 616–624 in the SERT protein backbone as an essential domain for vimentin association.

### Characterization of SITPET sequence of SERT

Inspection of the six amino acid difference between Δ20 and Δ14, the SITPET sequence, revealed 3 amino acids, S611, T613, and T616 as possible kinase action sites. We began to assess the effect of mutations of these 3 residues on uptake activity, whole cell, and surface expression. At each of the targeted locations, the original amino acid was changed to an alanine or aspartic acid (Fig. 5A).

**Figure 5:** *(A)* 5HT uptake rates of SITPET mutants. Twenty-four hour post-transfection CHO cells were washed and assayed for analysis of 5HT uptake rate. Background accumulation of (^3^H)-serotonin was measured in the same experiment using mock-transfected cells and subtracted from each experimental value. Maximum background accumulation was 0.01 pmol/mg protein/min. Phospho-mimicking mutations in the C-terminal region caused mixed results. The S_611_D mutation resulted in the most significant change over its neutral counterpart, S_611_A. Another key point is the drastic reduction seen when all 3 sites were mutated to aspartic acid and when only the two threonines were mutated to aspartic acid. Bars represent means±SD of three or more independent experiments. ANOVA indicated that the effect of the construct was highly significant (p<0.001). Multiple post-hoc comparisons versus control (SERT) were made applying Dunnett's correction; values marked with (**) were significantly different from control at p<0.05. Expression of SITPET mutants. The trafficking of mutants was assessed by gel electrophoresis and W/B. The detergent extracts of total protein were analyzed to determine if the alteration in uptake ability was due to alterations in the amount of protein. All variations of the transporter demonstrated similar protein expression levels. All lanes contain protein recovered from the same number of cells equivalent to 30% of one well from a confluent 24 well dish. The loading control was performed with actin (inset in the figure). The immunoblots are representative of at least three independently performed experiments. *(B)* Colocalization of YFP-SERT mutants on the plasma membrane. Cells were stained with Texas Red-WGA to mark the plasma membrane. The images show that DD and DDD mutations were totally retained on intracellular structures; S_611_D was found partially on the intracellular compartments. However, AAA and T_613_D were predominantly on the plasma membrane (arrowheads), but a pool of them resided on intracellular organelles. A 1 μm bar is presented for the image set.

A mutation to alanine is a relatively neutral change whereas a change to aspartic acid acts as a phospho-mimic at the site of mutation due to the charge and shape of the carboxylic acid functional group. 5HT uptake rates of each construct, S_611_A, T_613_A, T_616_A, and the triple mutation (AAA) retained 90, 74, 100 or 95% of the activity of wild-type transporter, respectively (Fig. 5A).

However, the single mutation of S_611_D caused a dramatic decrease in the uptake activity of SERT, reducing transport capacity to approximately 38%, whereas T_616_D caused no noticeable change in uptake function (Fig. 5A). Furthermore, the triple mutation to aspartic acid (DDD) caused a 95% reduction in the 5HT uptake capacity of SERT (Fig. 5A), possibly indicating a synergistic relationship between these three positions. In all cases, changes in transport capacity were not the result of altered protein expression levels, as indicated by W/B and densitometry analysis of total protein blots (Table 1).

**Table 1:** The whole cell expressions of all truncated and mutant forms of SERT in CHO cells were similar to those of the wild type transporter.

	SERT	Δ26	Δ20	Δ14	Δ6	S_611_A	S_611_D	T_613_A	T_613_D	T_616_A	T_616_D	AA	DD	AAA
**% of the total protein on the cell surface**	**80.33±5.5**	**0**	**0**	**65.3±2.5**	**65.3±2.3**	**70.6±3.05**	**30.6±1.53**	**54.33±4.04**	**55±4**	**79.6±0.58**	**79.6±0.58**	**78.6±3.2**	**8.3±2.9**	**99.3±1.15**
**5HT Uptake rates of transporters % of wild-type SERT**	**100**	**0**	**0**	**88**	**82**	**90**	**38**	**74**	**70**	**100**	**100**	**92**	**17**	**95**

The levels of transporter proteins on the plasma membrane were assessed by biotinylation of surface proteins followed by gel electrophoresis and W/B, and calculated as the percent of whole cell expression. The data presented in Table 1 are the average from three independent experiments, normalized as percentage of expression or 5HT uptake rates of wild-type transporter.

Investigation into the role of S611 in the 5HT uptake capacity of SERT was analyzed using the S_611_A and S_611_D constructs originally produced, while DD and AA, i.e., the double mutation of T613 and T616, were constructed to investigate the role of the two threonine residues in the proposed mechanism. S611 appeared to exert the most influence on the 5HT uptake rate of SERT.

Next, the expression of SITPET mutants on the plasma membrane was assessed by their colocalization with WGA, a plasma membrane marker (Fig. 5B). Mutants YFP-SERT variants were expressed in CHO cells and their distribution was compared with that of Texas Red conjugated wheat germ agglutinin, a lectin marker for the plasma membrane. The fluorescence data shown in Figure 5B indicate that the majority of DD and DDD were associated with intracellular structures. A significant part of AAA localized to the plasma membrane. Although a noteworthy pool of S611D appeared internally, some of S611D was observed on the plasma membrane (Fig. 5B).

In summary, DDD and DD were predominantly found at intracellular compartments while S_611_D located on the plasma membrane partially and mostly at intracellular compartments. Thus, the S_611_D transporter apparently has difficulties in membrane trafficking. In contrast, AAA and T_616_D were found on the plasma membrane (Fig. 5B and Table 1).

In an effort to explore the six amino acid difference between Δ20 and Δ14, the SITPET sequence, we began tested the association between endogenously expressed vimentin and transiently expressed mutant forms of transporters in 5HT-stimulated CHO cells with IP analysis (Fig. 6). The cellular proteins on the vimentin-Ab coated protein A beads were eluted and separated on SDS-PAGE followed by immunoblotting with SERT-Ab (Fig. 6). The major band at 90 kD was detected in the CHO-SERT, T_613_D, -T_616_D, and -AAA cells (Fig. 6). The 5HT uptake rates and the levels of surface expression of these forms were similar to the wild-type transporter (Fig. 5). Subsequently their levels of association with vimentin were high as well. On the other hand, the mutant that had a very minimal 5HT uptake rate and plasma membrane such as DDD did not associate with vimentin. Based on these findings, we hypothesize that the vimentin-binding ability of transporter is correlated with the density of transporter on the plasma membrane. In deed, S_611_D neither fully appeared on the plasma membrane, nor was pulled down by anti-vimentin antibody (Fig. 6). The 5HT uptake rate and the density of S_611_D on the plasma membrane (approximately 30% of the wild-type, Table 1) showed a similar pattern with its vimentin binding ability. The level of S_611_D precipitated on vimentin-Ab was 30% of the level of wild-type on vimentin-Ab.

**Figure 6:** Vimentin binding ability of SITPET mutants. CHO cells expressing the indicated SERT constructs were lysed and prepared for IP. The cell lysate was incubated with anti vimentin-Ab coated protein A sepharose beads. The presence of SERT truncations was detected with a polyclonal SERT Ab (Chemicon International). Nonspecific adsorption of Sepharose beads was not determined in the absence of vimentin-Ab and the data obtained from this set of experiment is not presented here since it can be found in Figure 1B. All lanes contain protein recovered from the same number of cells equivalent to one of well from a confluent 24-well culture plate. The triple mutant AAA and two of the single mutants, T_613_D and T_616_D, bound to vimentin; S_611_D showed a low affinity for binding to vimentin. Figure shows representative images from 3 separate experiments.

### Vimentin-SERT Association on the plasma membrane

Next, we evaluated the impact of 5HT stimulation on the density of truncated and mutant forms of transporters on the plasma membrane. CHO cells expressing Δ26, Δ20, Δ14, Δ6, S_611_D, T_613_D, T_616_D, AAA, and DDD were either directly (Fig. 7A, B ) or after stimulation with 100 μM 5HT (Fig. 7C, D) subjected to the cell surface biotinylation assay. Biotinylated membrane proteins were pulled down on streptavidin beads and eluted from the beads in SDS-PAGE sample buffer.

**Figure 7:** Impact of 5HT stimulation on the plasma membrane density of truncated and mutant transporters. CHO cells expressing truncated or mutant forms of transporter were either directly *(A and B)* or after stimulated with 100 μM 5HT *(C and D)* subjected to the cell surface biotinylation assays. Biotinylated membrane proteins were pulled down on streptavidin beads and eluted from the beads in SDS-PAGE sample buffer. The biotinylated eluents were subjected to immunoblot analysis using either anti-SERT *(A and C)*, or anti-vimentin *(B)*, or pS56-Ab *(D)*. All lanes contain protein recovered from the same number of cells equivalent to one of well from a confluent 24-well culture plate. In the surface protein experiments, we included two control experiments: mock biotinylated CHO cells transfected with SERT and mock transfected CHO cells. The first control, mock biotinylated CHO cells, were carried through the biotinylation procedure without the addition of the biotinylation reagent and neither of antibodies, SERT-, vimentin- nor pS56-Abs recognized proteins from these blots (data not presented). The next control, mock-transfected cells allowed us to observe (i) the nonspecific absorption of Sepharose beads and the proteins from the detergent soluble platelet lysate; (ii) if 5HT mediate any of these nonspecific interactions. Pretreatment with 100 μM 5HT increased the density of Δ14 and S_611_D, significantly or partially, respectively, and decreased the density of wild-type SERT and the truncated or mutant transporters which could to the plasma membrane. The transporters whose surface expressions were decreased with 5HT-stimulation, i.e., wild-type, Δ6, AAA, T_616_D, and T_613_D, were able to bind vimentin *(B)* and phosphovimentin *(D)*. However, the truncated or mutant forms transporters which could not bind vimentin *(B)* and appeared on the plasma membrane at high levels in 5HT-stimulation *(C)*, such as D14 and S_611_D, could not bind phosphovimentin *(D)*, either. The total phosphovimentin *(E)* and vimentin *(F)* (as flow through of the streptavidin beads) did not differ in truncated and mutant forms of transporter expressing CHO cells. The levels of vimentin and phosphovimentin in cell lysate of 100 mM 5HT-stimulated cells show if the associations between these proteins with SERT or truncated/mutant forms are altered with the differences in their levels, and/or with 5HT stimulation (Figure 7E and F). All lanes contain protein recovered from the same number of cells equivalent to 30% of one well from a confluent 24-well culture plate.

One half of the biotinylated membrane proteins were blotted with anti-SERT-Ab (Fig. 7A). Although there was some decrease in the densities of transporters on the plasma membrane of S_611_D transfected cells, Δ26, Δ20, and DDD were not located on the plasma membrane at all (Fig. 7A).

To evaluate the association of vimentin and the truncated and mutant transporters on the plasma membrane, the second half of the same biotinylated samples were subjected to immunoblot analysis with vimentin-Ab (Fig. 7B). In untransfected cells our W/B analysis recognized the endogenous vimentin as one of the proteins pulled by the biotinylated plasma membrane-bound proteins (Fig. 7B, the lane labeled as NoDNA). Therefore, it is clear that vimentin had bound other plasma membrane proteins as well as SERT.

In SERT transfected cells, the level of vimentin on the plasma membrane was much higher than the untransfected ones. This finding identifies SERT as one of the membrane-bound proteins that links vimentin to the plasma membrane. Similarly, the levels of vimentin on the plasma membrane of Δ26, Δ20, Δ14, and DDD transfected cells were the same as that on the plasma membrane of untransfected cells (Fig. 7B). This finding suggests a lack of association between vimentin and Δ26, Δ20, Δ14, or DDD on the plasma membrane. On the other hand, the vimentin-binding abilities of T_616_D and T_613_D on the plasma membrane were very similar to CHO-SERT and CHO-Δ6 cells.

The levels of vimentin on the plasma membrane of S_611_D transfected cells was lower than that in wild-type transfected cells but higher than that in untransfected ones. These findings are in good agreement with the data in Figure 6. Collectively, they support our hypothesis that the density of transporter on the plasma membrane and the level of its vimentin binding are correlated.

In summary, SERT is one of the proteins that link vimentin to the plasma membrane. Our co-IP studies in endogenous and heterologous expression systems, and IF analyses (Fig. 1, 3) demonstrate that in 5HT stimulated platelets the level of SERT precipitated on vimentin-Ab is higher than that in control platelets, which were altered by the extracellular level of 5HT.

We [15], [16] and others [11], [12] reported that 5HT stimulation at high levels does not increase the 5HT uptake rates and the density of SERT on the plasma membrane. Thus, we attempted to determine: (i) whether extracellular 5HT at high levels facilitates the translocation of SERT from the plasma membrane via phosphovimentin; and (ii) modification of three C-terminus residues, S_611_D, T_613_D, T_616_D, are involved in phosphovimentin-SERT association (Fig. 7C and D).

CHO cells expressing truncated and mutant forms of SERT were first stimulated with 100 μM 5HT, and then biotinylation assay was performed to separate the plasma membrane proteins and their partners. Biotinylated membrane proteins were pulled down on streptavidin beads and eluted from the beads in SDS-PAGE sample buffer.

One half of the biotinylated membrane proteins were blotted with anti-SERT-Ab (Fig. 7C). In agreement with reported studies, a pretreatment with 100 μM 5HT did not elevated the densities of SERT, Δ6, and the mutant transporters that mimic the phosphorylated forms, T_613_D and T_616_D, as 10 μM 5HT-stimulation did [15]. However, 5HT-stimulation increased the density of Δ14 truncated transporter and did not change the density of S_611_D mutant transporters on the plasma membrane (Fig. 7C).

In exploring the impact of phosphovimentin-SERT association on the plasma membrane density of SERT, the second half of the same biotinylated samples were subjected to immunoblot analysis with pS56, phosphovimentin-Ab (Fig. 7D). The data indicated that the association affinity between SERT and phosphovimentin on the plasma membrane was enhanced by 5HT stimulation.

The mutants, AAA, T_613_D, T_616_D, and the truncated form of the transporter, Δ6, which show decreased densities on the plasma membrane in response to 5HT stimulation, associated with phosphovimentin with high affinity (Fig. 7D). 5HT-stimulation does not alter the cell surface expression of S_611_D significantly or its association with phosphovimentin.

In these experiments, we included two control experiments: (i) mock biotinylated CHO cells transfected with SERT; and (ii) mock transfected CHO cells. The first control, mock biotinylated CHO cells, were carried through the biotinylation procedure without the addition of the biotinylation reagent and none of antibodies, SERT-, vimentin- nor pS56-Abs, recognized proteins from these blots (data not presented). The next control, mock-transfected cells, allowed us to observe (i) the nonspecific adsorption of Sepharose beads and the proteins from the detergent soluble platelet lysate; (ii) if 5HT mediate any of these nonspecific interactions.

The total phosphovimentin and vimentin (as flow through of the streptavidin beads) was similar between truncated and mutant forms of transporter expressing CHO cells (Fig. 7E and F).

The levels of vimentin and phosphovimentin in cell lysate of 100 mM 5HT-stimulated cells show if the associations between these proteins with SERT or truncated/mutant forms are altered with the differences in their levels, and/or with 5HT stimulation (Figure 7E and F).

Overall, these data suggest that the 5HT-dependent decrease in the surface expression of SERT directly correlates with its binding to phosphovimentin. Therefore, we hypothesize that in cells stimulated with a high level of 5HT, the surface density of SERT is decreased due to an increase in its association with phosphovimentin. In exploring this hypothesis, we tested the 5HT uptake rates and level of SERT on the cell surface in CHO cells transfected with 5HT-dependent phosphorylation site mutant vimentin, S56A and SERT.

### The impact of 5HT-stimulation on plasma membrane density of transporter

The amount of SERT on the plasma membrane is one of the important factors in determining the 5HT uptake rates of cells, which is controlled in a dynamic manner by the relative rates of transporter recycling from endosomes and internalization from the cell surface. In evaluating the role of phosphovimentin-SERT association on the surface expression of transporter, CHO cells co-expressing SERT and the vimentin S56A mutant were used in biotinylation assays followed by quantitative W/B either with SERT- or with pS56-Ab (Fig. 8A).

**Figure 8:** Effect of SERT-vimentin interaction on the surface expression of SERT. *(A)* CHO-SERT cells were pretreated with 0, 10, or 100 μM 5HT and biotinylated with NHS-SS-biotin (15, 16, 19). Biotinylated plasma membrane proteins were retrieved on streptavidin beads and analyzed for SERT or phosphovimentin- (pS56-) Ab by W/B. All lanes contain protein recovered from the same number of cells equivalent to one well from a confluent 24-well culture plate. *(B)* Intracellular SERT, vimentin, and phosphovimentin were also determined by W/B analysis of non-bound material. Mock-transfected CHO cells served as a control. Vimentin served as a loading control. The results of W/B analysis are the summaries of combined data from three densitometric scans. * represent differences from 0 μM 5HT-matched samples. All lanes contain protein recovered from the same number of cells equivalent to 30% of one well from a confluent 24-well culture plate. *(C)* CHO cells expressing SERT and phosphovimentin mutant S56A were first pretreated with (0–100 μM) 5HT, and then their 5HT uptake rates were measured in intact cells as described under “Materials and Methods.” Background accumulation of (^3^H)-serotonin was measured in the same experiment using mock-transfected cells and subtracted from each experimental value. Maximum background accumulation was 0.01 pmol/mg protein/min. Rate of uptake is expressed as the means and SD values of triplicate determinations from three independent experiments. ANOVA indicated that the interaction between 5HT level and cell line was highly significant (p<0.001) for both figures (B and C). Post-hoc comparisons were adjusted using a Bonferroni correction. Significant comparisons with the uptake rates of mock transfected CHO cells within 5HT level are indicated with *, and with 0 μM 5HT within cell line are indicated with # (all p≤0.001).

The plasma membrane density of SERT in CHO-SERT cells stimulated with 100 μM 5HT appeared lower than in cells stimulated with 10 μM 5HT. The quantification of these data is summarized in Table 2.

**Table 2:** Effect of 5HT pretreatment on SERT Expression.

Percent change of SERT in 5HT pretreated cells compare to untreated cells				
	CHO-SERT	CHO-(SERT+S56A)	CHO-SERT	CHO-(SERT+S56A)
	SERT expression on cell membrane		SERT expression in cell lysate	
**10 μM (5HT)_ex_**	44.4% ↑	47% ↑	35% ↓	35% ↓
**100 μM (5HT)_ex_**	5.7% ↓	40% ↑	5% ↑	No change

In CHO-SERT and CHO-(SERT+S56A) cells, the effect of 5HT pretreatment on the surface density of SERT proteins was tested at two different concentrations: at low (10 μM) and high (100 μM) 5HT. Twenty-four hour post-transfected cells were pretreated with 5HT and biotinylated with NHS-SS-biotin [18], [23], [26]. Intracellular SERT and biotinylated plasma membrane proteins were analyzed with W/B with SERT antibodies. The results of W/B analysis are the summary of combined data from three densitometric scans denoted as the percent change of SERT density in 5HT pretreated cells compared to untreated cells.

Stimulation with 10 μM 5HT increased the density of SERT on the plasma membrane of CHO-SERT cells 44.4%, whereas 100 μM 5HT stimulation did not show this enhancement on the density of SERT on the plasma membrane compared to untreated CHO-SERT cells. At high concentrations, 5HT stimulation reduced the plasma membrane density of SERT and resulted in a loss of uptake function in platelet system (30%) that was more severe than that in the heterologous system (5.7%). Apparently, these differences are due to the factors involved in the translocation of SERT from/to the plasma membrane, which are either not found in endogenous and heterologous expression systems equally, or the expressions levels in both systems are not stochiometrically sufficient to play their roles correctly.

Additionally, the immunoblots revealed that in cells stimulated with 100 μM 5HT, the transporters bound significant amounts of phosphovimentin on the plasma membrane (Fig. 8A).

Next, we tested the impact of SERT-phosphovimentin association on the plasma membrane density of SERT. CHO cells were co-transfected with SERT and pS56A constructs, stimulated with 10 or 100 μM 5HT, and then subjected to cell surface biotinylation. Immunoblots of the biotinylated membrane proteins demonstrated that in the absence of phosphovimentin, 100 μM 5HT-stimulation kept the plasma membrane density of SERT at the level found in 10 μM 5HT-stimulated levels (Fig. 8A and B).

We wanted to follow up these findings by correlating the biochemical characteristics of CHO-(SERT+pS56A) cells with their 5HT uptake measurement (Fig. 8C). Cells co-expressing the phosphorylation mutant form of vimentin, pS56A and transporter, did not reveal the wild-type phenotype of 5HT-downregulated 5HT uptake. In this respect, they behaved identically to the cells stimulated with 10 μM 5HT.

## Discussion

The plasma membrane level of SERT is altered by the rate of the translocation transporter protein to/from the plasma membrane which is controlled through its interaction with other proteins in these pathways. It was well documented that the plasma level of 5HT plays a role in the density of SERT on the plasma membrane via PKC-mediated phosphorylation of SERT [12], [22]. Additionally, the C-terminus region of SERT is vital to the ability of these transporters to function [14]. Our studies here identify a novel pathway by correlating how plasma 5HT plays a role on the translocation of SERT from the plasma membrane via using the C-terminus region of transporter.

The density of SERT on the plasma membrane is modulated by its interaction with other proteins such as an adaptor protein, Hic-5 plays a role in the internalization of SERT in platelets [13]. Also, the C-terminal region of SERT was identified as a domain of interaction with the actin cytoskeleton [8]. Relevant findings include that the C-terminal of SERT interacts with MacMARCKS, a substrate of PKC that binds to the actin cytoskeleton, and the fact that PKC modulators, such as β-PMA, modulate the activity of SERT [8], [10], [11], [23]. Our data further support this contention by demonstrating that C-terminal truncated forms of SERT show a loss of functional membrane trafficking. This loss of function may relate to the level of interact between SERT and cytoskeleton network.

Our studies with SERT in transient transfection systems reveal that the truncation of various lengths of the C-terminus altered the 5HT uptake rate of SERT transporters. Truncation of the final 26 and 20 amino acid residues of SERT completely abolished uptake, whereas truncation of the final 14 and 6 residues resulted in a 12% to 18% loss in transport capacity as compared to full length SERT. These results agree with published reports for NET and SERT [14], [24, respectively], which demonstrate that truncation of the C-terminus abolished the uptake rates of these transporters. However, a single residue removal from the C-terminus of NET caused a 60% reduction in uptake capacity [24]. Here, we demonstrate that truncation of the final 14 residues of SERT resulted in a transporter that still retained approximately 90% of its 5HT uptake rate.

Further analysis of the difference between Δ20 and Δ14 truncations of the SERT C-terminus, which retained 0% compared to 90% transport rates, respectively, revealed the sequence SITPET. Within this region, there are 3 potential phosphorylation sites at S611, T613, and T616. Several studies have demonstrated that PKC modulators, such as βPMA, reduce SERT localization on the plasma membrane and blunt 5HT uptake capacity [1], [11], [12], [22], [23], [25]–[28]. Additionally, these studies also established an interaction of PP2A, a component of the protein phosphatase complex, with SERT [29]–[31]. Based on these findings, we analyzed the effects of phosphorylation-mimicking amino acids on the 5HT uptake rate of SERT. Our results indicate that S611 may be a key site for phospho-regulation, since the single mutation of S611 to D caused a 61% decrease in 5HT uptake rate whereas the single mutation of S611 to A caused no reduction in 5HT uptake. T613 and T616 individually do not appear to be critical phospho-regulatory residues since neither mutation (A or D) of T613 and T616 showed a similar level of 5HT uptake rate. However, it is possible that these sites work in conjunction with each other to modulate the function of the transporter since our results indicate that the triple mutation DDD of 611, 613, and 616 retained only 5% of its 5HT uptake capacity as compared to control SERT. It is also important to note that the presence of such a large amount of negative charge on the end of the protein could cause alterations in protein folding or protein-protein associations that are important for protein function, resulting in the observed blunting of transport capacity.

Next, we analyzed the impact of four truncations of the SERT C-terminus on the trafficking and expression of SERT on the plasma membrane using biotinylation and IF assays. Our data indicate that depending on the amount of truncation from the C-terminus of SERT, there was altered localization of the transporter. Therefore, we carried out a biotinylation analysis on some of the phosphorylation-mimicking mutations in an effort to determine the plasma membrane localization of these mutants, i.e., whether the mutation arrests them intracellularly or whether the mutants can still traffic to the plasma membrane. The data indicate that 3 possible phosphorylation sites do contribute to the 5HT uptake rates of transporters via inhibiting their proceedings toward the plasma membrane. The proteins involved in the membrane trafficking of SERT are still under investigation by many laboratories.

Our biochemical and proteomic analysis of the platelet proteins associated with the C-terminus of SERT demonstrate an association between vimentin, an intermediate filament, and SERT in platelets. Association also was noted in a CHO heterologous expression system. Vimentin is the major type III intermediate filament expressed in cells of mesenchymal (*e.g.* endothelium, fibroblasts, megakaryocytes) and myogenic origin [32]. Vimentin, a minor component of the platelet cytoskeleton [33], is associated with the Triton X-100 insoluble fraction of human platelets [34], [35]. Studies have shown that vimentin forms a network of intermediate filaments that form a ring close to the cell membrane, as well as a network that activates PAK-dependent phosphorylation of vimentin, altering the filamentous structure of this cytoskeletal compound. Our studies demonstrate an association between vimentin and SERT in the cytosol and on the plasma membrane of platelet and CHO-expression system within 5HT-independent manner. Collectively, these findings point to vimentin as a possible candidate for facilitating the translocation of SERT between intracellular compartments and plasma membrane. When 5HT-stimulation dependent phosphorylation was eliminated, the surface expression and the 5HT uptake rates of SERT were restored in CHO cells treated with 100 μM 5HT. Of the several C-terminus mutant transporters, only Δ14 and S_611_D did not associate with vimentin although both could appear on the plasma membrane in active form. Additionally, neither the plasma membrane expressions of these two mutant transporters were decreased in 100 μM 5HT-treated cells, nor they were able to bind phosphovimentin. These data strengthen our hypothesis that the modification of the SITPET sequence differentially, one amino acid at a time, exposes the vimentin binding domain on the C-terminus of SERT. However, elevated plasma 5HT controls the cellular distribution of SERT on an “altered” vimentin network, the translocation of SERT from the plasma membrane is accelerated on the 5HT-altered vimentin network. Thus, in plasma of hypertensive subjects in which 5HT reaches a high level, the platelet SERT may continue to clear plasma 5HT with a lower Vmax, most likely until the plasma 5HT levels come back to the physiological level [16].

Therefore, to the best of our knowledge, this is the first study to identify a sequence on the C-terminus of SERT that regulates the rate of 5HT uptake by altering the density of SERT on the plasma membrane via differential phosphorylation of SITPET sequence, which facilitates the association of SERT with an intermediate filament, vimentin.

Recent investigations indicate a system of phosphorylation for SERT that incorporates two phases of phosphorylation [11]. The first phase of phosphorylation is said to affect the serine residues, whereas the second phase involves the threonine residues. It is suggested that the first phase of phosphorylation causes the transporters to shut down, and the second phase of phosphorylation tags the proteins for internalization via the SERT recycling mechanism. According to the biphasic model, a S_611_D construct should shut down the uptake ability of the transporter while the DD construct should demonstrate a reduced or eliminated 5HT uptake capacity due to its intracellular localization. Indeed, our data agree with the study by Jayanthi et al. [11], who reported that S_611_D reduces transport capacity by ∼39%, whereas DD (T613+T616) demonstrates an uptake capacity of ∼16%. On the basis of our findings, we hypothesize that the blunted activity (∼39%) of S_611_D may be due to additional serine residues that play a role in reducing the uptake capacity of SERT. A finding that was not consistent with the biphasic theory was the localization of S_611_D, which is mainly found at intracellular locations.

In summary, in an endogenous platelet system and in heterologous expression systems, our studies demonstrate that vimentin associates with SERT. The last 20 amino acids from the C-terminus of SERT are required and are at least one of the binding-domain(s) of vimentin. SERT becomes a bridge between vimentin and the plasma membrane. At physiological plasma 5HT levels, vimentin-SERT association was found at intracellular locations and on the plasma membrane (Fig. 7B). However, when plasma 5HT level was higher than physiological level, their association was enhanced and the level of SERT on the plasma membrane was decreased. Therefore, we hypothesize that SERT utilizes the vimentin network during translocation from the plasma membrane. Furthermore, the 5HT-dependent phosphorylation of vimentin on the S56 residue accelerates the translocation of SERT on the 5HT-altered vimentin network. Future analysis of these mutants in stable transfection systems, as well as continued experiments with the phospho-mimicking mutants presented here, will further reveal the mechanism of action that governs transporter C-terminal phosphorylation. These studies also will advance our understanding of the specific processes by which phosphorylation of the C-terminus plays a role.

## Supporting Information

Table S1 (0.03 MB PDF)
